RETRACTED

# Naringin Promotes Osteogenic/Odontogenic Differentiation of Dental Pulp Stem Cells via Wnt/*β*-Catenin

**DOI:** 10.1155/2022/4505471

**Published:** 2022-05-29

**Authors:** Meiling Guo, Fen Liu, Wenjuan Wang, Zhirong Liu, Zhipeng Zhu, Yiyu Liu, Zhen Huang

**Affiliations:** ^1^Department of General Dentistry, The Affiliated Stomatological Hospital of Nanchang University, Nanchang City, Jiangxi Province 330006, China; ^2^The Key Laboratory of Oral Biomedicine, Nanchang City, Jiangxi Province 330006, China; ^3^Jiangxi Province Clinical Research Center for Oral Diseases, Nanchang City, Jiangxi Province 330006, China; ^4^Department of Orthodontics, The Affiliated Stomatological Hospital of Nanchang University, Nanchang City, Jiangxi Province 330006, China

## Abstract

**Purpose:**

This investigation intended to unravel the effect and mechanism of naringin on the proliferation and osteogenic differentiation of human dental pulp stem cells (hDPSCs).

**Methods:**

hDPSCs were induced to differentiate, and the degree of cell differentiation was observed by alizarin red staining, Oil Red O staining, and Alcian blue staining. hDPSCs were treated with 0, 20, 40, and 80 *μ*mol/L naringin for 48 h, respectively. The proliferation rate and chemotaxis of the cells were measured by MTT and transwell assay, alkaline phosphatase (ALP) activity and osteogenic differentiation degree by ALP staining and alizarin red staining, and gene expression of osteogenic markers by qRT-PCR. Additionally, western blot was performed to test the levels of Wnt/*β*-catenin signaling-related proteins in hDPSCs.

**Results:**

The isolated hDPSCs with spindle-shaped morphology had good differentiation capability. Further experiments confirmed naringin-caused increases in the proliferation rate and migration ability of hDPSCs. In addition, compared with the control group, naringin-treated cells had strong ALP activity and ossification levels and higher expression of Runx2, OPN, DSPP, and DMP1. The western blot results showed that naringin significantly activated Wnt/*β*-catenin signaling in hDPSCs.

**Conclusion:**

Taken together, naringin enhances the proliferation, migration, and osteogenesis of hDPSCs through stimulating Wnt/*β*-catenin signaling pathway.

## 1. Introduction

The advent of regenerative medicine provides the opportunities to regenerate and repair human organs, becoming a significant contributor to clinical treatment [1]. Stem cells are a key resource in regenerative medicine, which are clonogenic and self-renewing progenitor cells with the ability to generate into one or more specialized cell types [2]. Mesenchymal stem cells (MSCs) are a kind of adult stem cells with capacity for self-renewal and multilineage differentiation, so they have emerged as a seed cell source for tissue regeneration and tissue engineering [3]. Human dental pulp stem cells (hDPSCs) are one type of MSCs present in the cell-rich zone and core of the dental pulp, resembling characteristics of MSCs [4]. hDPSCs can repair injured tissue and promote the proliferation and regeneration of dentin-pulp [5]. Collectively, hDPSCs can also be an important cell source applied in regenerative medicine. However, *in vitro* stem cell culture has always been a difficult problem, and hDPSC culture is no exception. Such problem seriously affects the application and promotion of stem cells, so it is essential to seek new growth factors for inducing cell stemness.

RETRACTED

Naringin is the main flavonoid compound extracted from tomatoes, grapefruit, and citrus fruits, and flavonoids are the secondary metabolites and the source of bioactive compounds in plants [6]. An extensive literature survey has presented that naringin possesses antioxidant, anti-inflammatory, antiapoptotic, antiulcer, antiosteoporosis, and anticarcinogenic properties [7]. Further in-depth study has proved naringin can affect cell differentiation and proliferation through improving signal transduction pathway activity. It enhances the activity of UMR-106 cells via inhibition of HMG-CoA reductase [8] and can regulate the PI3K/AKT signaling pathway to increase the expression of bone morphogenetic protein-2, osteopontin and osteoprotegerin, and osteocalcin [9]. Additionally, naringin promotes bone morphogenetic protein secretion in bone marrow mesenchymal stem cells (BMSCs) and enhances cell proliferation and osteogenic differentiation [10]. In the study by Cao et al., naringin depresses NF-*к*B signaling pathway activity to achieve the rescue of TNF-*α*-induced inhibition of osteogenesis of BMSCs [11]. In human adipose-derived mesenchymal stem cells (hADMSCs), naringin activates the Wnt signaling to protect the cells from hydrogen peroxide-induced oxidative stress and inhibition of osteogenic differentiation [12]. *In vivo*, naringin can significantly enhance the bone regeneration ability of mice, and at the same time, no obvious toxicity and side effects were found at the dose of 400 mg/kg [13]. The above findings are good evidence that naringin has a mighty growth-promoting function for cell development and inhibits apoptosis and aging in *C. elegans* [14, 15]. However, there is no relevant study on the effect of naringin on the proliferation and differentiation of hDPSCs. This study therefore set out to explore the effects of naringin on chemotaxis and osteogenic differentiation of hDPSCs and determine whether the potential mechanism is related to Wnt/*β*-catenin signaling pathway. Drawing upon the following experiments, we attempt to provide a new method and data basis for *in vitro* culture of DPSCs.

RETRACTED

## 2. Materials and Methods

### 2.1. Cell Culture and Cell Processing

hPDLSCs were obtained from American Type Culture Collection (ATCC) and cultured in ɑ-MEM medium (Gibco, USA) containing 10% fetal bovine serum (FBS; Gibco, USA) at 37°C in a 5% CO_2_ incubator. The cell culture medium was changed every 3 days.

hDPSCs were divided into four groups and received intervention of 0 *μ*mol/L naringin (control group), 20 *μ*mol/L naringin (NRG-L group), 40 *μ*mol/L naringin (NRG-M group), and 80 *μ*mol/L naringin (NRG-H group), respectively. After 48 hours of intervention, the plates were collected for the following experiments.

### 2.2. Induction of Dental Pulp Stem Cell Differentiation

hDPSCs were seeded onto the 6-well plates at a density of 2 × 10^4^ cells/mL. The corresponding medium was prepared for induction of osteogenic, adipogenic, and chondrogenic differentiation. For osteogenic induction, the medium was added osteogenic induction solution containing 0.1 *μ*mol/L dexamethasone, 50 *μ*mol/L vitamin C, and 10 mmol/L *β*-glycerophosphate and changed every three days; the cells were differentiated and matured after 14 days of culture. For adipogenic induction, the induction solution was supplemented with 1 *μ*mol/L indomethacin, 0.5 mmol/L IBMX, 10 *μ*g/mL insulin, removed after 3 days; the cells were differentiated and matured after 12 days, and the lipid droplet formation was observed by Oil Red O staining. For chondrogenic differentiation, the cells were digested with trypsin and then 1 mL of 2 × 10^5^ cells/mL cell suspension was added to a 15 mL centrifuge tube (1000 r/min, 3 min). After centrifugation, the cells were transferred to a medium with addition of 10 *μ*g/mL ITS-X, 10 ng/mL LTGF-*β*3, 1.0 *μ*g/mL dexamethasone, and 5.35 *μ*g/mL linoleic acid; the cells were differentiated and matured after 4 weeks, and the chondrogenic state of the cells was observed by Alcian blue staining.

### 2.3. Detection of Surface Antigens of Human Dental Pulp Stem Cells

The first passage of isolated hDPSCs was digested with 0.25% trypsin and counted, with the cell density adjusted to 1 × 10^6^ cells/mL. The antibodies of hDPSC surface-related antigens (CD45, CD90, CD34, and CD73) were diluted in precooled PBS buffer according to the instructions and then added into the cells and incubated for 1 h in the dark. After that, the cells were washed three times with precooled PBS. Finally, they were detected by flow cytometry and were examined using a microscope for morphology.

RETRACTED

### 2.4. MTT Assay

hDPSCs in the logarithmic growth phase after treatment were seeded in 96-well plates at a density of 100 cells/well and cultured for 24 h, 48 h, and 72 h, respectively. Then, 20 *μ*L of 5 mg/mL MTT solution was added to each group of cells and cultured for another 4 h in the incubator. After the supernatant was aspirated, the samples were added with 150 *μ*L of DMSO and then shaken for 15 min. Absorbance at 570 nm was determined using a microplate reader.

### 2.5. Transwell Assay

First, 100 *μ*L of cell suspension was seeded in the upper chamber, with 700 *μ*L of medium containing 20% fetal bovine serum in the lower chamber. Transwell inserts were taken out after 12–24 h of incubation at 37°C with 5% CO_2_, washed three times with PBS, and then fixed in 1% glutaraldehyde for 30 min. Subsequently, on completion of PBS rinsing and drying, the cells were stained with 0.1% crystal violet for 12 h and washed in PBS and dried again. Six to ten visual fields were randomly observed under an inverted microscope to count the positive cells in each field. Finally, three fields were randomly selected for photography and statistical analysis.

### 2.6. Alkaline Phosphatase (ALP) Staining and ALP Activity Assay

On day 7 of inducing osteogenic differentiation, the culture medium of hDPSCs in each group was removed. Then, they were washed three times with PBS solution at 37°C and fixed in 4% paraformaldehyde for 30 min. After removing the fixation solution, three PBS washes were carried out. Next, the cells were stained with the BCIP/NBT ALP staining kit and incubated for 30 min away from light. After removing the staining solution, three PBS washes were performed and the staining was observed. The ALP activity of the cells was assessed using an ALP activity assay kit (Nanjing Jiancheng Bioengineering Institute, China) according to the manufacturer's instructions.

### 2.7. Alizarin Red Staining

On day 21 of inducing osteogenic differentiation, the culture medium of hDPSCs in each group was removed. Then, they were washed three times with PBS solution at 37°C and fixed in 4% paraformaldehyde for 15 min. After removing and three PBS washes, each well was added moderate 2% alizarin red staining solution and incubated for 15 min at room temperature. The formation of mineralized nodules was observed after removing the staining solution and three PBS washes again.

### 2.8. qRT-PCR

The total RNA of cells in each group was extracted using the TRIzol method. Subsequently, the concentration and purity of RNA were detected by NanoDrop and cDNA was prepared according to the random primer reverse transcription kit (Thermo, USA). The mRNA expression levels of Runx2, OPN, DSPP, and DMP1 were detected according to the instructions of the SYBR GREEN kit (Takara, Japan), and GAPDH was used as the internal reference. Six replicates were set up in the experiment. The relative expression of the target gene was calculated by the 2^−ΔΔCt^ method. Primer sequences are shown in Table 1.

RETRACTED

### 2.9. Western Blot

The whole proteins of cells were extracted by RIPA buffer, and the concentration of extracted proteins was quantified using a BCA kit. Subsequently, 20 *μ*g of protein with 1 × loading buffer was boiled for denaturation. Proteins were isolated using sulfate-polyacrylamide gel electrophoresis (SDS-PAGE) and then transferred to polyvinylidene fluoride (PVDF) membrane. Next, the membrane was blocked using 5% skim milk powder for 1 h and incubated overnight at 4°C with primary antibodies. Then, the membrane was rinsed three times prior to and after another 1 h incubation with secondary antibodies at ambient temperature. The proteins were visualized using enhanced chemiluminescence reagent, and the pictures were collected by the gel imaging system. The gray levels of bands were quantified using ImageJ software with GAPDH as an internal reference for relative protein expression analysis.

### 2.10. Statistical Analysis

SPSS 25.0 was used for one-way analysis of variance (ANOVA) and independent-samples *t*-test analysis. The outcomes were expressed as mean ± standard deviation (SD). The statistical significance was assumed when *p* < 0.05.

## 3. Results

### 3.1. Phenotype and Characterization of Human Dental Pulp Stem Cells

The flow cytometry results showed the negative results of hDPSC surface antigens CD34 and CD45 and positive results of CD73 and CD90 (Figure 1(a)). Additionally, the cells presented with spindle-shaped morphology under a microscope (Figure 1(b)). The results of different differentiation of cells indicated that mineralized nodules were observed after osteogenic differentiation, intracellular lipid droplets were observed after adipogenic differentiation, and blue chondroid matrix deposition was observed after chondrogenic differentiation (Figures 1(c)–1(e)).

### 3.2. Naringin Promotes the Proliferation and Chemotaxis of Human Dental Pulp Stem Cells

The results of MTT assay presented that the proliferation rate of hDPSCs treated with naringin was significantly increased compared with the control group and naringin concentration was positively correlated with the proliferation rate (Figure 2(a)). Transwell assay for investigating the effect of naringin on chemotaxis of hDPSCs revealed that the NRG-M group and NRG-H group notably enhanced the chemotaxis of hDPSCs in the control group (Figures 2(b) and 2(c)).

RETRACTED

### 3.3. Naringin Promotes the Osteogenic Ability of Human Dental Pulp Stem Cells

The results of ALP staining and ALP activity assay of hDPSCs in the control, NRG-L, NRG-M, and NRG-H groups are shown in Figures 3(a) and 3(b). In comparison with the control group, naringin remarkably increased ALP activity in hDPSCs and the increase was in a concentration-dependent manner. Furthermore, the alizarin red staining results suggested that the mineralization level of hDPSCs gradually increased in the naringin-treated groups in a concentration-dependent manner (Figures 3(c) and 3(d)). The gene expression of osteogenic markers Runx2, OPN, DSPP, and DMP1 also had an increase after naringin treatment according to qRT-PCR results (Figures 3(e)–3(h)).

### 3.4. Naringin Activates the Wnt/*β*-Catenin Signaling Pathway

To clarify the mechanism of naringin promoting osteogenic differentiation of hDPSCs, we examined the levels of Wnt/*β*-catenin signaling pathway-related proteins by western blot analysis. To be specific, naringin increased the protein levels of Wnt3a, *β*-catenin, CyclinD1, and p-GSK-3*β* in hDPSCs in a concentration-dependent manner in comparison with the control group (Figures 4(a) and 4(b)).

## 4. Discussion

Dental pulp is an unmineralized oral tissue occupying the central pulp cavity of each tooth, which is composed of soft connective tissue and vascular, lymphatic, and neural elements [16]. hDPSCs are ectodermal-derived stem cells originating from migrating neural crest cells [17]. They have MSC properties and fibroblast-like morphology, seeded onto plastic surfaces and forming colonies after *in vitro* culture [17]. hDPSCs with multilineage differentiation potential can differentiate into chondrocytes, adipocytes, odontoblast-like cells, and neural-like cells under appropriate induction [18]. A previous study uncovered that BMSCs had a higher lineage potential to differentiate into cartilage and bone compared with ADMSCs [19], and DPSCs are superior to BMSCs in proliferation rate, colony formation ability, and mineralization potential [20]. Liu et al. reported that DPSCs expressed a range of mesenchymal markers (CD29, CD44, CD59, CD73, CD90, and CD146) and did not express hematopoietic markers (CD34, CD45, and CD11b) [21]. In our experiment, the isolated hDPSCs exhibiting spindle morphology had good potential of osteogenic, adipogenic, and chondrogenic differentiation and their surface antigens CD90 and CD73 were positive, while CD45 and CD34 were negative. Collectively, we successfully isolated hDPSCs.

hDPSCs are promising in the field of regenerative medicine and have been applied in research studies regarding pancreatic, cardiac, and cornea reconstruction. DPSCs can secrete proangiogenic and antiapoptotic factors to repair drug-induced myocardial infarction in nude rats [22]. Monteiro et al. confirmed that tissue-engineered DPSCs were successfully transplanted to reconstruct the corneal epithelium in an animal model with limbal stem cell deficiency [23]. These suggest that DPSCs can play a pivotal role in regenerative medicine and provide a window in the untapped potential of these cells. Nevertheless, most MSCs are relatively difficult to obtain and culture *in vitro*, resulting in some limitations in the clinical application [24] and greatly hindering the development of regenerative medicine. In the existing studies, DPSCs were treated with dentin matrix components to promote their differentiation into dentin [25] or were stimulated by eight small molecule complexes such as valproic acid to enhance neurogenic differentiation and maturation [26]. Resveratrol can also increase the expression of the neuron-specific marker genes (Nestin, Musashi, and NF-M) in DPSCs and induce cell differentiation into neurons [27]. In this study, we used naringin to promote the proliferation and chemotaxis of hDPSCs, improve their osteogenic and odontogenic ability, and upregulate the gene expression levels of osteogenic markers.

RETRACTED

Wnt signaling is involved in processes essential for embryonic development and homeostasis in normal adults. The Wnt/*β*-catenin signaling pathway is universally associated with differentiation, cell polarity, and migration [28], and it has been proved to play a vital role in the regulation of MSC differentiation [29, 30]. This pathway is activated during the stem cell definitive stage while inhibited at osteoblast maturation [31]. Naringin has strong potential to promote cell proliferation and differentiation, and its effect is achieved through the Wnt/*β*-catenin signaling pathway. For example, in hip arthroplasty, naringin enhances osteoprotegerin expression through the Wnt/*β*-catenin signaling pathway in fibroblasts from periprosthetic membrane [32]. Also, it promotes the mRNA and protein expressions of *β*-catenin and improves Ser552 phosphorylation on *β*-catenin in UMR-106 cells, leading to the activation of lymphoid enhancer factor/T-cell factor transcription factors and thereby improving skeletal development [33]. In our study, naringin also activated the Wnt/*β*-catenin signaling pathway. Collectively, naringin exerts its biological function through the Wnt/*β*-catenin signaling pathway.

## 5. Conclusion

In summary, naringin activates the Wnt/*β*-catenin signaling pathway to promote the proliferation and chemotaxis of hDPSCs and their osteogenic and odontogenic ability. In clinical practice, DPSCs are usually cultured *in vitro* and then transplanted into the body, but the problem of *in vitro* culture of DPSCs has been difficult to solve. The above results illustrate that naringin is a growth-promoting factor facilitating *in vitro* DPSC culture and provides more possibilities for the application and promotion of stem cell transplantation therapy. Naringin is therefore a natural substance worthy of utilization by regenerative medicine. However, this study is still limited in the investigation of molecular mechanism of naringin stimulating Wnt/*β*-catenin signaling. Further exploration is needed to provide a more comprehensive data basis for clinical application of naringin.

RETRACTED

## Figures and Tables

**Figure 1:** Phenotype and characterization of human dental pulp stem cells. (a) Flow cytometry was used to detect the expression of hDPSC surface antigens (CD34, CD45, CD73, and CD90). (b) Cell morphology of hDPSCs was observed under a light microscope. (c) Cellular lipid synthesis was examined using Oil Red O staining. (d) Mineralized nodules were viewed by alizarin red staining. (e) Chondroid matrix deposition was observed by ALP staining.

**Figure 2:** Naringin promotes the proliferation and chemotaxis of human dental pulp stem cells. (a) MTT assay was employed for measuring the cell proliferation in the control, NRG-L, NRG-M, and NRG-H groups. (b, c) Chemotaxis of hDPSCs verified by transwell assay in each group. ^*∗*^*p* < 0.05 and ^*∗∗*^*p* < 0.01 vs. control group; ^##^*p* < 0.01 vs. NRG-L group; ^i÷i÷^*p* < 0.01 vs. NRG-M group.

**Figure 3:** Naringin promotes the osteogenic ability of human dental pulp stem cells. (a, b) ALP staining and activity assays of hDPSCs after 7 days of osteogenic induction. (c, d) Alizarin red staining and quantitative outcomes of mineralized nodules of hDPSCs after 21 days of osteogenic induction. (e–h) qRT-PCR assay of Runx2, OPN, DSPP, and DMP1 expression in hDPSCs. ^*∗∗*^*p* < 0.01 vs. control group; ^##^*p* < 0.01 vs. NRG-L group; ^i÷i÷^*p* < 0.01 vs. NRG-M group.

**Figure 4:** Naringin activates the Wnt/*β*-catenin signaling pathway. (a, b) Western blot assay of Wnt3a, *β*-catenin, CyclinD1, and p-GSK-3*β* expression in hDPSCs. ^*∗∗*^*p* < 0.01 vs. control group; ^#^*p* < 0.05 and ^##^*p* < 0.01 vs. NRG-L group; ^i÷i÷^*p* < 0.01 vs. NRG-M group.

**Table 1:** Primer sequences.

RNA	Sequences (5′ to 3′)
Runx2	F: 5′-CCCAGTATGAGAGTAGGTGTCC
	R: 5′-GGGTAAGACTGGTCATAGGACC

OPN	F: 5′-TCTGCTACCTCCAAGTGTGGCT
	R: 5′-GCAGTATGCGAAGACCATCACC

DSPP	F: 5′-CAACCATAGAGAAAGCAAACGCG
	R: 5′-TTTCTGTTGCCACTGCTGGGAC

DMP1	F: 5′-GAGCAGTGAGTCATCAGAAGGC
	R: 5′-GAGAAGCCACCAGCTAGCCTAT

GAPDH	F: 5′-CATCACTGCCACCCAGAAGACTG
	R: 5′-ATGCCAGTGAGCTTCCCGTTCAG

RETRACTED

## Data Availability

The data presented in this article are available on request.

## References

[1] Sedgley CMBotero T. M. (2012). Dental stem cells and their sources. *Dental Clinics of North America*.

[2] Rodriguez-Lozano F. J., Bueno C., Insausti C. L. (2011). Mesenchymal stem cells derived from dental tissues. *International Endodontic Journal*.

[3] Suchanek J., Soukup T., Ivancakova R., Karbanova J., Hubkova V., Pytlik RKucerova L. (2007). Human dental pulp stem cells—isolation and long term cultivation. *Acta Medica*.

[4] Gridly M. M., Abbass M. G., Abdel-Hafez AMMokhtar N. M. (1989). Effect of antidepressant “Parnate” on salivary glands and dorsal surface of the tongue of albino rats, Histological and histochemical study. *Egyptian Dental Journal*.

[5] Sonoda S., Mei Y. F., Atsuta I. (2018). Exogenous nitric oxide stimulates the odontogenic differentiation of rat dental pulp stem cells. *Scientific Reports*.

[6] Bacanl M., Baaran AABaaran N. (2018). The major flavonoid of grapefruit: naringin. *Polyphenols: Prevention and Treatment of Human Disease*.

[7] Burke A. C., Sutherland B. G., Telford D. E., Morrow M. R., Sawyez C. G., Edwards JYHuff M. W. (2019). Naringenin enhances the regression of atherosclerosis induced by a chow diet in Ldlr(-/-) mice. *Atherosclerosis*.

[8] Bharti S., Rani N., Krishnamurthy BArya D. S. (2014). Preclinical evidence for the pharmacological actions of naringin: a review. *Planta Medica*.

[9] Yin F. M., Xiao LBZhang Y. (2015). Research progress on Drynaria fortunei naringin on inflammation and bone activity. *Zhong Guo Gu Shang*.

[10] Zhang P., Dai K. R., Yan S. G. (2009). Effects of naringin on the proliferation and osteogenic differentiation of human bone mesenchymal stem cell. *European Journal of Pharmacology*.

[11] Cao X., Lin W., Liang C. (2015). Naringin rescued the TNF-*α*-induced inhibition of osteogenesis of bone marrow-derived mesenchymal stem cells by depressing the activation of NF-*к*B signaling pathway. *Immunologic Research*.

[12] Wang L., Zhang Y. G., Wang X. M., Ma LFZhang Y. M. (2015). Naringin protects human adipose-derived mesenchymal stem cells against hydrogen peroxide-induced inhibition of osteogenic differentiation. *Chemico-Biological Interactions*.

[13] Chen L. L., Lei L. H., Ding P. H., Tang Q., Wu Y. M. (2011). Osteogenic effect of Drynariae rhizoma extracts and Naringin on MC3T3-E1 cells and an induced rat alveolar bone resorption model. *Archives of Oral Biology*.

[14] Zhao H., Liu M., Liu H., Suo R., Lu C. (2020). Naringin protects endothelial cells from apoptosis and inflammation by regulating the Hippo-YAP Pathway. *Bioscience Reports*.

RETRACTED

[15] Zhu Q., Qu Y., Zhou X. G., Chen J. N., Luo H. R., Wu G. S. (2020). A dihydroflavonoid naringin extends the lifespan of *C. elegans* and delays the progression of aging-related diseases in PD/AD models via DAF-16. *Oxidative Medicine and Cellular Longevity*.

[16] Gronthos S., Mankani M., Brahim J., Robey PGShi S. (2000). Postnatal human dental pulp stem cells (DPSCs) in vitro and in vivo. *Proceedings of the National Academy of Sciences of the U S A*.

[17] Ranganathan KLakshminarayanan V. (2012). Stem cells of the dental pulp. *Indian Journal of Dental Research*.

[18] Martens W., Bronckaers A., Politis C., Jacobs RLambrichts I. (2013). Dental stem cells and their promising role in neural regeneration: an update. *Clinical Oral Investigations*.

[19] Li MIkehara S. (2013). Bone-marrow-derived mesenchymal stem cells for organ repair. *Stem Cells International*.

[20] Alge D. L., Zhou D., Adams L. L. (2009). Donor-matched comparison of dental pulp stem cells and bone marrow-derived mesenchymal stem cells in a rat model. *Journal of Tissue Engineering and Regenerative Medicine*.

[21] Liu J., Yu F., Sun Y. (2015). Concise reviews: characteristics and potential applications of human dental tissue-derived mesenchymal stem cells. *Stem Cells*.

[22] Gandia C., Arminan A., Garcia-Verdugo J. M. (2008). Human dental pulp stem cells improve left ventricular function, induce angiogenesis, and reduce infarct size in rats with acute myocardial infarction. *Stem Cells*.

[23] Monteiro B. G., Serafim R. C., Melo G. B. (2009). Human immature dental pulp stem cells share key characteristic features with limbal stem cells. *Cell Proliferation*.

[24] Gu Y., Bai YZhang D. (2018). Osteogenic stimulation of human dental pulp stem cells with a novel gelatin-hydroxyapatite-tricalcium phosphate scaffold. *Journal of Biomedical Materials Research Part A*.

[25] Alongi D. J., Yamaza T., Song Y. (2010). Stem/progenitor cells from inflamed human dental pulp retain tissue regeneration potential. *Regenerative Medicine*.

[26] Heng B. C., Jiang S., Yi B., Gong T., Lim LWZhang C. (2019). Small molecules enhance neurogenic differentiation of dental-derived adult stem cells. *Archives of Oral Biology*.

[27] Geng Y. W., Zhang Z., Liu MYHu W. P. (2017). Differentiation of human dental pulp stem cells into neuronal by resveratrol. *Cell Biology International*.

[28] Duchartre Y., Kim Y. M. (2016). The Wnt signaling pathway in cancer. *Critical Reviews in Oncology*.

[29] Glass D. A., Karsenty G. (2007). In vivo analysis of Wnt signaling in bone. *Endocrinology*.

[30] Xiang L., Zheng J., Zhang M., Ai TCai B. (2020). FOXQ1 promotes the osteogenic differentiation of bone mesenchymal stem cells via Wnt/*β*-catenin signaling by binding with ANXA2. *Stem Cell Research & Therapy*.

RETRACTED

[31] Valenti M. T., Dalle Carbonare LMottes M. (2016). Osteogenic differentiation in healthy and pathological conditions. *International Journal of Molecular Sciences*.

[32] Yang C., Liu W., Zhang X., Zeng BQian Y. (2020). Naringin increases osteoprotegerin expression in fibroblasts from periprosthetic membrane by the Wnt/*β*-catenin signaling pathway. *Journal of Orthopaedic Surgery and Research*.

[33] Wang D., Ma W., Wang F., Dong J., Wang D., Sun B. (2015). Stimulation of wnt/*β*-catenin signaling to improve bone development by naringin via interacting with AMPK and akt. *Cellular Physiology and Biochemistry*.

